This article has been retracted.

# Smartphone Interventions Effect in Pediatric Subjects on the Day of Surgery: A Meta-Analysis

**DOI:** 10.3389/fsurg.2021.759958

**Published:** 2021-12-16

**Authors:** Li Li, Jianping Ma, Dan Ma, Xiaokang Zhou

**Affiliations:** ^1^Department of Pediatrics, Hebei Children's Hospital, Shijiazhuang, China; ^2^Department of Pediatric Orthopedics, Hebei Children's Hospital, Shijiazhuang, China; ^3^Operating Room, The Third Hospital of Shijiazhuang City, Shijiazhuang, China; ^4^Department of Pediatric Orthopedics, Hebei Children's Hospital, Shijiazhuang, China

**Keywords:** pediatric, surgery, anxiety at induction, smartphone interventions, oral midazolam, modified Yale Preoperative Anxiety Scale

## Abstract

**Background:** A meta-analysis was performed to evaluate the effect of smartphone interventions on the anxiety of the pediatric subjects at induction on the day of surgery compared to oral midazolam or standard care as control.

**Methods:** A systematic literature search up to June 2021 was performed and nine studies selected 785 pediatric subjects on the day of surgery at the start of the study; 390 of them were using smartphone interventions, 192 were control, and 203 were using oral midazolam. They were reporting relationships between the effects of smartphone interventions on the anxiety of the pediatric subjects at induction on the day of surgery compared to oral midazolam or control. The mean difference (MD) with its 95% CIs was calculated to assess the effect of smartphone interventions on the anxiety of the pediatric subjects at induction on the day of surgery compared to oral midazolam or control using the continuous method with a fixed or a random-effects model.

**Results:** Smartphone interventions in pediatric subjects were significantly related to lower anxiety at induction on the day of surgery (MD, −19.74; 95% CI, −29.87 to −9.61, *p* < 0.001) compared to control and significantly related to lower anxiety at induction on the day of surgery (MD, −7.81; 95% CI, −14.49 to −1.14, *p* = 0.02) compared to oral midazolam.

**Conclusion:** Smartphone interventions in pediatric subjects on the day of surgery may have lower anxiety at induction compared to control and oral midazolam. Further studies are needed to confirm these findings.

## Background

Based on the previous studies, the more anxious a child is before surgery, the more possible they will be to experience delirium and progress to negative postoperative behavior (1, 2). Also, children might have sleeping difficulties (1), fears, and eating difficulties after surgery (3). The hospitalized children families similarly notice high levels of stress and anxiety (4, 5). Children are influenced by distress of the families (1, 6, 7). It may influence both the negative and positive emotional state for families, if their children are going to surgical management (8). A pain management at home after day surgery is similarly significant, since most children are rated as suffering from significant pain on the 2nd day following surgery (1, 9). One way to decrease the anxiety of child or pain is to use distraction, which can shift their attention to something else apart from the anxiety and pain (10, 11). Distraction is used as a non-pharmacological pain technique used by families and health professionals. Distractions are both active and passive. For children, active distractions comprise the use of interactive toys, virtual reality, guided imagery, controlled breathing, and relaxation. Passive distractions comprise watching television, videos, and listening to music (10–12). Comedy or therapeutic play is a good active distraction for children, since this could decrease their anxiety before surgery (13, 14). One additional example of such distraction is medical clowns or clown therapy (15–17). Clown therapy is not probable to use or might not be cost-effective. So, it is vital to discover cost-effective techniques, e.g., web-based smartphone interventions. Smartphone health is a new area of healthcare that could be used for enabling subjects and their families in self-care (18–20). Smartphone apps or games could be used as active or passive distractions and could decrease anxiety and pain in children and their families in surgery situations. Web-based smartphone interventions are typically psychologically based and delivered by the smartphone platforms and the Internet (21, 22). Technological innovations are quickly developing; we have an increasing number of smartphone apps and games that children could use for distraction while waiting for surgery. It was previously shown effective to let children play an interactive video game while getting the anesthetic by the facemask (23). It was considered as a better distraction than the oral midazolam or the attendance of the families at the surgery (23). Furthermore, earlier studies have reported that smartphone applications decrease the perioperative anxiety of the children (24, 25). It was also found that an interactive distraction such as playing video games helps children in handling acute pain than a passive distraction, e.g., watching videos while children had a cold pressor. This study aimed to evaluate the effect of smartphone interventions on the anxiety of the pediatric subjects at induction on the day of surgery compared to oral midazolam or control.

## Methods

This study completed here followed the meta-analysis of studies in the epidemiology statement (26), following an established protocol.

### Study Selection

Studies comprised were that stated statistical measures of relationship [odds ratio (OR), mean difference (MD), frequency rate ratio, or relative risk, with 95% CIs] measuring the effect of smartphone interventions on the anxiety of the pediatric subjects at induction on the day of surgery compared to oral midazolam or control.

Only human studies in the English language were selected. Inclusion was not limited by study type or size. Excluded studies were commentary and review articles and articles did not provide a degree of association. Figure 1 shows the whole study process.

**Figure 1:** Diagram of the study process.

Articles, included in our meta-analysis, had to meet the following inclusion criteria:

1. This study should be prospective or retrospective.
2. The target population is pediatric subjects on the day of surgery
3. The intervention program was the smartphone interventions, oral midazolam, and standard care as control.
4. This study comprised comparisons between the effects of smartphone interventions on the anxiety of the pediatric subjects at induction on the day of surgery and oral midazolam or standard care as control. The level of the anxiety of the pediatric subjects at induction was measured using the modified Yale Preoperative Anxiety Scale.

The exclusion criteria were:

1. Studies that did not compare smartphone interventions to oral midazolam or standard care as control.
2. Studies with a condition other than on the day of surgery.
3. Studies did not focus on the influence of comparative results.

### Identification

A search protocol strategies were prepared according to the PICOS principle (27) as follow: P (population): pediatric subjects on the day of surgery; I (intervention/exposure): smartphone interventions; C (comparison): effect of smartphone interventions on the anxiety of the pediatric subjects at induction on the day of surgery compared to oral midazolam or control; O (outcome): children anxiety at induction; and S (study design): no restriction (28). First, a systematic search was conducted by OVID, Embase, Cochrane Library, PubMed, and Google Scholar, from January 2012 to January 2021, using a mixture of keywords and similar words for pediatric surgery, anxiety at induction, smartphone interventions, oral midazolam, and the modified Yale Preoperative Anxiety Scale as shown in Table 1. Selected studies were collected in an EndNote file, duplicates were omitted, and the titles and abstracts were reviewed to remove studies that did not report the association between the effects of smartphone interventions on the anxiety of the pediatric subjects at induction on the day of surgery compared to oral midazolam or control based on the previously mentioned exclusion and inclusion criteria. The remaining articles were revised for associated information.

**Table 1:** Search strategy for each database.

**Database**	**Search strategy**
Pubmed	#1 “pediatric surgery”[All Fields] OR “anxiety at induction”[All Fields] #2 “smartphone interventions”[MeSH Terms] OR “pediatric”[All Fields] OR “oral midazolam”[All Fields] OR “modified Yale Preoperative Anxiety Scale”[All Fields] #3 #1 AND #2
Embase	'pediatric surgery'/exp OR 'anxiety at induction'/exp #2 'smartphone interventions'/exp OR 'ICBG'/exp OR 'oral midazolam' OR 'modified Yale Preoperative Anxiety Scale' #3 #1 AND #2
Cochrane library	#1 (pediatric surgery):ti,ab,kw OR (anxiety at induction):ti,ab,kw (Word variations have been searched) #2 (smartphone interventions):ti,ab,kw OR (oral midazolam):ti,ab,kw OR (modified Yale Preoperative Anxiety Scale):ti,ab,kw (Word variations have been searched) #3 #1 AND #2

### Screening

Data were abbreviated based on the following; study-related and subject-related features onto a homogeneous form as follow; the primary author last name, study period, country, publication year, the studies region, and type of the population, design of the study; and the total number of subjects, demographic data, and clinical and treatment features. In addition, the evaluation period associated with measurement, quantitative method and qualitative method of assessment, source of information, outcomes assessment, and statistical analysis MD or relative risk, with 95% CI of relationship (29). If a study is suitable for inclusion based upon the above principles, data were extracted separately by the two authors. In case of inconsistency, the corresponding author gave a final choice. When there were various data from a study, the data were extracted individually. There is a risk of bias (RoB) in these studies; therefore, individual studies were evaluated using two authors who independently assessed the methodological quality of the selected studies. The “RoB tool” from the RoB 2: a revised Cochrane RoB tool for randomized trials was utilized to evaluate methodological quality (30). In terms of the evaluation criteria, each study was evaluated and allocated to one of the next three RoB—low: if all the quality criteria were met, the study was considered to have a low RoB; unclear: if one or more of the quality criteria were partially met or unclear, the study was considered to have a moderate RoB; or high: if one or more of the criteria were not met or not included, the study was considered to have a high RoB. Any discrepancies were addressed by a reassessment of the original article.

### Eligibility

The main result focused on measuring the effect of smartphone interventions on the anxiety of the pediatric subjects at induction on the day of surgery compared to oral midazolam or control. Evaluation of the measurement of the effect of smartphone interventions on the anxiety of the pediatric subjects at induction on the day of surgery compared to oral midazolam or control was extracted forming a summary.

### Inclusion

Sensitivity analyses were restricted only to studies showing a relationship among the effect of smartphone interventions on the anxiety of the pediatric subjects at induction on the day of surgery compared to oral midazolam or control. For subcategory and sensitivity analysis, the effect of smartphone interventions compared to that of oral midazolam or control was used.

### Statistical Analysis

We determine the MD and 95% CI using the continuous technique with a fixed-effect model or a random-effect model. We determined the *I*^2^ index, which was between 0 and 100%. When the *I*^2^ index was about 0, 25, 50, and 75%, it identifies no, low, moderate, and high heterogeneity, respectively (27). We used a random-effect model if the *I*^2^ was > 50%; we used a fixed-effect model if the *I*^2^ was < 50%. We stratified the original evaluation per outcome categories as described before to complete the subgroup analysis. A *p*-value for differences between subcategories of < 0.05 was considered as statistically significant. Publication bias was evaluated quantitatively using the Egger's regression test (publication bias is existing if *p* ≥ 0.05) and qualitatively by visual examination of funnel plots of the logarithm of ORs against their standard errors (29). The whole *p*-values were two-tailed. The Reviewer Manager version 5.3 (The Nordic Cochrane Center, The Cochrane Collaboration, Copenhagen, Denmark) was used to do all the calculations and graphs.

## Results

A total of 534 unique studies were selected, of which nine studies (between 2012 and 2021) satisfied the inclusion criteria and were comprised in this study (31–39).

The nine studies included 785 pediatric subjects on the day of surgery at the start of the study; 390 of them were using smartphone interventions, 192 were control, and 203 were using oral midazolam. All the studies evaluated the effect of smartphone interventions on the anxiety of the pediatric subjects at induction on the day of surgery compared to oral midazolam or control.

Study size ranged from 64 to 115 pediatric subjects on the day of surgery at the start of this study. The details of the nine studies are shown in Table 2. Five studies reported data stratified to smartphone interventions compared to control and four studies stratified to smartphone interventions compared to oral midazolam.

**Table 2:** Characteristics of the selected studies for the meta-analysis.

**References**	**Country**	**Total**	**Web-based smartphone intervention**	**Control**	**Oral midazolam**
Mifflin et al. (31)	Canada	89	42	47	
Kerimoglu et al. (32)	USA	64	32	32	
Seiden et al. (33)	USA	108	57		51
Fortier et al. (34)	USA	82	38	44	
Marechal et al. (35)	France	115	60		55
Stewart et al. (36)	USA	102	51		51
Al-Nerabieah et al. (37)	Syria	64	32	32	
Uyar et al. (38)	Turkey	91	45		46
Jung et al. (39)	USA	70	33	37	
	**Total**	**785**	**390**	**192**	**203**

Smartphone interventions in pediatric subjects were significantly related to lower anxiety at induction on the day of surgery (MD, −19.74; 95% CI, −29.87 to −9.61, *p* < 0.001) with high heterogeneity (*I*^2^ = 94%) compared to control as shown in Figure 2 and significantly related to lower anxiety at induction on the day of surgery (MD, −7.81; 95% CI, −14.49 to −1.14, *p* = 0.02) with high heterogeneity (*I*^2^ = 84%) compared to oral midazolam as shown in Figure 3.

**Figure 2:** Forest plot of the outcome of smartphone interventions compared to control on anxiety at induction on the day of surgery.

**Figure 3:** Forest plot of the outcome of smartphone interventions compared to oral midazolam on anxiety at induction on the day of surgery.

Selected studies do not provide a layered analysis tailored to the types of surgery, age, and ethnicity, as no study reported or adjusted these factors.

Based on the visual inspection of the funnel plot and quantitative measurement using the Egger's regression test, there was no evidence of publication bias (*p* = 0.87). However, most of the included studies were assessed to be of low methodological quality due to their small sample size. All the studies did not have selective reporting bias and no articles had incomplete outcome data and selective reporting.

## Discussion

Smartphone interventions in the pediatric subjects may have lower anxiety at induction on the day of surgery compared to control or oral midazolam (31–39). However, the analysis of results should be done with caution due to the low number of studies in the present meta-analysis and the low sample size of most of the selected studies (ix out of nine studies were < 100), proposing the requirement for additional studies comparing smartphone interventions to control or oral midazolam in the pediatric subjects on anxiety at induction on the day of surgery to validate these findings.

The studies involved in our meta-analysis evaluated the effect of web-based smartphone interventions on the pediatric subjects on the day of surgery. The interventions comprised active and passive distractions, e.g., videos or gaming smartphone apps, with games that are age-appropriate and easily accessible on the Internet (31–33, 35, 36). Web-based smartphone interventions custom-made and that are educational for pediatrics will be required due to the hospital care digitalization. This will decrease the dependence of the children on the capability of their families to prepare them on the day of the surgery. All the smartphone interventions needed Internet access. The challenge here is the availability of such interventions for all the pediatric subjects because a smartphone or an iPad is essential to take benefit of these smartphone interventions. Most people have their smartphones, but there are subjects groups whose socioeconomic condition might affect their use of the smartphone intervention. Kerimoglu et al. have shown that there was a weak relation between heart rate and the modified Yale Preoperative Anxiety Scale; heart rate was possibly not a precise secondary measure of anxiety in the preoperative situation (32). Studies of earlier web-based smartphone interventions varied in their intervention types and result measures (24, 25, 40). Chow et al. found that audiovisual interventions decreased the anxiety of children (41).

There is a little proof that web-based smartphone interventions decrease pain of the pediatric subjects in a postoperative situation. Though, in all the studies, the surgery types were variable. This may result in variations of postoperative pain. Pain levels in pediatric patients were determined in one study (42); it was stated that it would be important to examine postoperative pain and the possibility of analgesics administration at home. In a meta-analysis of audiovisual smartphone interventions by Chow et al., postoperative pain was determined in two studies, which increases the requirement for additional studies on postoperative pain in web-based smartphone interventions (41).

This meta-analysis reported the association between smartphone intervention use and their effects on the anxiety of the pediatric subjects at induction on the day of surgery. However, more studies are needed to validate these probable relations. Moreover, more studies are needed to supply a clinically meaningful difference of the outcomes in pediatric subjects on the day of surgery. These studies must comprise larger homogeneous samples. This was suggested similarly in an earlier similar meta-analysis study, which reported a comparable effect of smartphone interventions, oral midazolam, and control in pediatric subjects on the day of surgery (43). Also, another meta-analysis of audiovisual interventions suggested the need for a study to cover different age and surgery types (41). Well-conducted studies are furthermore needed to assess these factors and the mixture of different types of surgery, age, and ethnicity; since our meta-analysis study could not answer whether they are associated with the results. In summary, the data recommend that smartphone interventions in the pediatric subjects on the day of surgery may have lower anxiety at induction compared to control or oral midazolam. Further studies are needed to confirm these findings (44).

## Limitations

There might be selection bias in this study since several selected studies were excluded from the meta-analysis. However, the excluded studies did not satisfy the inclusion criteria of our meta-analysis. Similarly, whether the outcomes are related to the type of surgery, age, and ethnicity or not could not be answered. The study designed to assess the relationship between the effects of smartphone interventions on the anxiety of the pediatric subjects at induction on the day of surgery compared to oral midazolam or control was based on data from earlier studies, which may result in bias persuaded by incomplete details. The meta-analysis was based on a small number of studies (nine studies); six studies were small < 100. Variables including the type of surgery, ethnicity, and nutritional status of subjects were also the possible bias-inducing factors. Some unpublished articles and missing data may cause a bias in the pooled result. Subjects were using different management schedules and healthcare systems. There is a risk of language bias, since we only incorporated studies in English. In some studies, the authors reported a robust method of collecting the data: the anxiety levels were collected by reliable psychologists. In other studies, anxiety of the children was determined by healthcare staff, which may have influenced the heterogeneity.

## Conclusion

Smartphone interventions in the pediatric subjects may have lower anxiety at induction on the day of surgery compared to control and oral midazolam. Further studies are required to validate these findings. However, the analysis of results should be done with caution due to the low number of studies in the present meta-analysis and the low sample size of most of the selected studies, proposing the requirement for additional studies comparing smartphone interventions to control or oral midazolam on the anxiety of the pediatric subjects at induction on the day of surgery to validate these findings.

## Data Availability Statement

The original contributions presented in the study are included in the article/supplementary material, further inquiries can be directed to the corresponding author/s.

## Author Contributions

LL and JM contributed to the planning, data entry, and writing. DM contributed to the planning statistics and writing. XZ contributed to the concept, planning of study design, statistics, and writing. All authors contributed to the article and approved the submitted version.

## Conflict of Interest

The authors declare that the research was conducted in the absence of any commercial or financial relationships that could be construed as a potential conflict of interest.

## Publisher's Note

All claims expressed in this article are solely those of the authors and do not necessarily represent those of their affiliated organizations, or those of the publisher, the editors and the reviewers. Any product that may be evaluated in this article, or claim that may be made by its manufacturer, is not guaranteed or endorsed by the publisher.
